This article has been retracted.

# Considering Computational Mathematics IGHG3 as Malignant Melanoma Is Associated with Immune Infiltration of Malignant Melanoma

**DOI:** 10.1155/2022/4168937

**Published:** 2022-04-18

**Authors:** Mengqing Si, Xianwei Cao

**Affiliations:** ^1^Queen Mary College, Medical Department, Nanchang University, Nanchang, China; ^2^The Second Affiliated Hospital of Nanchang University, Nanchang, China; ^3^Department of Dermatology, The First Affiliated Hospital of Nanchang University, Nanchang, China

## Abstract

Malignant melanoma is one of the most threatening cancers to human health. Only 14% of patients with malignant melanoma have a remaining life span of 5 years. At present, there have been some studies looking for potential prognostic indicators of esophageal cancer from the level of genes and infiltrating immune cells, but there are still some problems that need to be resolved urgently. This paper proposes IGHG3 as the immune infiltration of malignant melanoma, which takes into account the computational mathematics. It aims to deduce the characteristics of immune cell infiltration in malignant melanoma and study the relationship between different immune cell infiltration characteristics and prognosis. The method in this article is to establish a computational mathematical model for the immunotherapy of melanoma, then study the method of identification of the affinity of the IGHG3 reagent, and finally obtain the gene expression of immune infiltration. The functions of these methods are, respectively, to predict the dynamic behavior of T cells with two different specificities through mathematical models and to test the matching degree of different concentrations of IGHG3 reagent with the human body. Then use the ssGSEA algorithm to obtain immune infiltration related data and calculate the difference between the weighted empirical cumulative distribution function of all genes in the effect of IGHG3 on melanoma that was carried out. The experimental results showed the computational mathematical method genome and all the remaining genes. In this study, a computational mathematical method to detect the IGHG3 gene expression had a significant inhibitory effect on A375 cells in the experimental group, and the knockdown efficiency reached 85.6%.

## 1. Introduction

Malignant melanoma has a high incidence and a high mortality rate. There are no special clinical symptoms in the early stage of onset, so it is found relatively slowly and the prognosis is poor. Melanoma is more harmful to patients than ordinary cancer. It can lead to rapid death of patients, and melanoma can bring a series of adverse symptoms to patients. A popular research direction in cancer research is the study of immune infiltration. Cancer progression and prognosis are strongly related to different levels of immune cell infiltration. In this paper, through the gene discovery matrix, the content and types of immune cells in a variety of tissues can be estimated and the general methods include valuation method and CIBERSORT. Therefore, studying malignant melanoma cells from the perspective of genetics and finding effective biological targets is an important method to improve the diagnosis rate of early malignant melanoma. At the same time, effective biological targets can also provide new clinical ideas for the treatment and prognosis of melanoma. Therefore, a thorough investigation of potential immunotherapy targets is very important for developing target drugs and improving the cure rate of cancer.

The main treatment options for malignant melanoma are surgery, chemotherapy, radiation therapy, biological therapy, etc. These treatment methods have very limited effects on malignant melanoma. Therefore, seeking new treatments is very important for patients with malignant melanoma, and immune infiltration is a very practical idea. Through some gene matrix data research, this article directly calculates the content of immune cells and extracts these content through complex experiments. This study constructed a prognostic model from different perspectives of the biological characteristics of melanoma and integrated it into the nomogram model, in order to predict the prognosis of patients with malignant melanoma more accurately. The results of this study have improved the accuracy of individualized predictions and treatment options for patients. IGHG3 can be supplemented outside of surgery, using high-dose IGHG3 inhibitors combined with MEK inhibitors, but this treatment has no evidence-based medical evidence and application experience.

Melanoma has gradually become a major obstacle to human health, so more and more scholars are exploring ways to cure the disease. Weinan believes that computational mathematics based on neural networks can approximate very high-dimensional functions with unprecedented efficiency and accuracy. This is not only in the field of traditional artificial intelligence, but also in the fields of scientific computing and computational science. He described some of the most important progress made on these issues, hoping to put things in perspective that would help to combine machine learning with computational mathematics [1]. Carette believes that SageMath is now a complete computational mathematics system. This system is used by many researchers and is increasingly used in classrooms. Computational mathematics is SageMath's strong point. He pays close attention to this point. His research covers algebra/analysis, numerical calculation, and combination [2, 3]. Mokrani proposed the ABCD (asymmetric, irregular border, color, and dermoscopic structure) rule of dermoscopy as a scoring method used by dermatologists to quantify the results of dermoscopy and effectively distinguish melanoma from benign lesions. He implemented automatic ABCD scoring of dermoscopy lesions and proved through experiments that the algorithm achieved a sensitivity of 91.25% and a specificity of 95.83% [4]. Cui's research aims to explore the functional role of miR-301a in melanoma and its possible molecular mechanism. He found that the expression of miR-301a in melanoma tissues was significantly increased, and the increase of miR-301a was related to the metastasis and prognosis of melanoma patients [5]. Han proposed that surgery is the main treatment for malignant melanoma of the rectum. However, whether the abdominal perineal resection is to remove a local tumor or a large tumor is still a controversial issue. He studied 4 patients with malignant melanoma of the rectum who underwent laparoscopic abdominal perineal resection, and the long-term follow-up results of these patients were relatively good [6]. Sheng aims to describe gene expression profiles related to PD-1 and its ligands PD-L1 and PD-L2 and then to decrypt their probabilistic biological processes in melanoma. He studied the relationship between PD1/PD-L1/PD-L2 and immune infiltration and checkpoints through expression analysis and also analyzed the role of PD-1/PD-L1/PD-L2 in determining clinical results [7]. Yenerall analyzed the status of NSCLC cell lines after receiving clinically relevant chemotherapy, targeted inhibitors or radiotherapy, combined with highly specific RUVBL1/2 inhibitors or their enantiomer controls, and measured the cells vitality [8]. He concluded that RUVBL1/2 inhibited melanoma cells, but could not significantly enhance the killing effect of chemotherapy or other targeted drugs. In addition, in vitro treatment of NSCLC with RUVBL1/2 inhibitors and radiation will activate the cGAS/STING pathway, indicating that RUVBL1/2 inhibitors can be combined with radiation and immunotherapy [9]. Vadakekolathu aims to study the immune status of characterizing mutant AML and determine whether TP53 abnormalities may use an investigative bispecific dual affinity and retargeting antibody (DART) molecule to immunotherapy patients [10].

In this study, the author obtained the gene performance data and clinical data of malignant melanoma, the data comes from the TCGA database, then calculate the ratio of various immune cells in melanin tissue and normal tissue samples, and use CIBERSORT software and mathematical algorithms to analyze the relationship between immune cell infiltration and the patient's tumor stage and prognosis. The CIBERSORT software uses the method of deconvolution and uses the data of a single cell to extract the features and inversely infer the proportions of various cell components.

## 2. Methods of Immune Infiltration of Malignant Melanoma

### 2.1. The Computational Mathematical Model of Melanoma Immunotherapy

In this paper, the generalized continuation theorem Lyapunov function method and the principle of differential equation comparison in the theory of coincidence degree are used to discuss the dynamic properties of several types of biological models, including the existence and uniqueness of periodic solutions, the sufficient conditions for the existence of multiple periodic solutions, and the existence and global stability of asymptotically periodic solutions. The initial mathematical model of tumor immunotherapy considered three groups of cancer cells, immune executive cells, and IL-2 neurons. The model is expressed as

(1) $$\begin{array}{c} \left\{\begin{array}{c} \frac{dx\left(n\right)}{dt}=cy\left(n\right)-\mu_{2}x\left(n\right)+\frac{p_{2}x\left(n\right)z\left(n\right)}{g_{1}+z\left(n\right)}+s_{1},\\ \frac{dy\left(n\right)}{dt}=r_{2}y\left(n\right)\left(1-by\right.\left(n\right)-\frac{ax\left(n\right)z\left(n\right)}{g_{2}+y\left(n\right)},\\ \frac{dz\left(n\right)}{dt}=\frac{p_{2}x\left(n\right)y\left(n\right)}{g_{3}+y\left(n\right)}-\mu_{3}z\left(n\right)+s_{2}. \end{array}\right. \end{array}$$

The initial conditions are

(2) $$\begin{array}{c} x\left(n\right)=x_{0},y\left(n\right)=y_{0},z\left(n\right)=z_{0}. \end{array}$$

The number of immune executive cells, the number of cancer tumor cells, and the number of IL-2 cell divisions are represented, respectively. The coefficient of anti-tumor performance is expressed by parameter C, the proliferation rate of tumor cells is expressed as, the reduction rate of IL-2 is expressed as, and a is the intensity of immune response [11]. S1 and S2, respectively, represent the amount of immune executive cells and locus IL-2 imported from the patient's body during treatment. The other parameters are constants. At the same time, a 3-dimensional tumor model with immune response and chemotherapy is used. Numerical simulation and optimal control theory prove that when the chemical reaction occurs instantaneously, the solution of the system when the drug is added is close to the solution of the system without drug treatment [12]. The specific model is as follows:

(3) $$\begin{array}{c} \left\{\begin{array}{c} \frac{dN\left(n\right)}{dt}=r_{2}N\left(n\right)\left(1-b_{2}N\left(n\right)\right)-c_{4}T\left(n\right)N\left(n\right)-a_{3}\left(1-e^{-u}\right)N\left(n\right)\\ \frac{dT\left(n\right)}{dt}=r_{1}T\left(n\right)\left(1-b_{1}T\left(n\right)\right)-c_{2}T\left(n\right)I\left(n\right)-c_{3}T\left(n\right)N\left(n\right)-a_{2}\left(1-e^{-u}\right)T\left(n\right) \end{array}.\right. \end{array}$$

The number of normal cells, the number of cancerous tumor cells, and the number of immune-reactive cells are, respectively, indicated as one of them. Therefore, this experiment established a model of melanoma skin cancer based on this model:

(4) $$\begin{array}{c} \left\{\begin{array}{c} n_{x}=n_{x}\left(b\right.\left(x\right)-d\left(x\right)-c\left(x,y\right)n_{y}-s\left(x,x\right)-s_{w}\left(x,x\right)n_{w}\\ n_{y}=n_{y}\left(b\right.\left(y\right)-d\left(y\right)-c\left(y,x\right)n_{y}-s\left(y,x\right)+s_{w}\left(y,x\right)n_{x} \end{array}\right.. \end{array}$$

Among them are the number of differentiated melanoma cells and the number of dedifferentiated melanomas [13]. The parameters represent the birth rate and mortality of differentiated melanoma cancer cells and represent the core competition between differentiated melanoma cells and dedifferentiated melanoma cells. But because in the final experimental results, T cells cannot kill dedifferentiated melanoma cancer cells; therefore, this article proposes to establish two types of T cells in future treatments, which can recognize and kill differentiated melanoma cells and dedifferentiated melanoma cancer cells, respectively [14]. Based on this hypothesis, this paper uses a mathematical model to predict the kinetic behavior of T cells with two different specificities for treatment, and a model can be established:

(5) $$\begin{array}{c} \left\{\begin{array}{c} n_{zx}=n_{zx}\left(b\left(z_{x},x\right)n_{x}-d\left(z_{x}\right)\right)\\ n_{zy}=n_{zy}\left(b\left(z_{y},y\right)n_{y}-d\left(z_{y}\right)\right) \end{array}.\right. \end{array}$$

Among them, it means two types of T cells can recognize differentiated melanoma cells and dedifferentiated melanoma cells [15, 16]. The model proposed above is simplified below, and the material exchange between cells is shown in Figure 1.

The simplified model is

(6) $$\begin{array}{c} \left\{\begin{array}{c} \frac{dM}{dt}=\left(b_{m}-d_{m}\right)M-s_{MD}M+s_{DM}D\\ \frac{dD}{dt}=\left(b_{D}-d_{D}\right)D+s_{MD}M-s_{DM}D \end{array}\right.. \end{array}$$

Here the natural birth rate of T cells is set to 0 because they are produced by adoptive cell transfer and will not proliferate without a target [17]. In order to avoid the uncertainty of the problem, this article introduces new parameters. These two parameters, respectively, represent the net growth rate of the two tumor cells. This can simplify the original model and reduce the number of parameters [18]. After introducing new parameters, the above model can be transformed into

(7) $$\begin{array}{c} \left\{\begin{array}{c} \frac{dM}{dt}=T_{M}M-s_{MD}M+s_{DM}D\\ \frac{dD}{dt}=R_{d}D+s_{MD}M-s_{DM}D \end{array}\right.. \end{array}$$

### 2.2. IGHG3 Reagent Affinity Identification Method

The ELISA method uses the specific reaction of the antigen and the antibody to connect the test substance and the enzyme, and then the enzyme and the substrate produce a color reaction for quantitative determination. The target of the measurement may be an antibody or an antigen. In this study, the indirect ELISA method was used to determine the affinity constant (Ka) of the IGHG3 reagent antibody. Using Pb2 + -ITCBE-BSA with concentrations of 1.0 mg/L, 2.0 mg/L, and 4.0 mg/L to dilute the known concentration of Pb2 + Mab by multiples. The dilution levels are as follows: 6 *μ*g/mL, 3 *μ*g/mL, and 1.5 *μ*g/mL, following the indirect ELISA method to determine the A450nm value of each well. The horizontal axis is mAb concentration, the vertical axis is A450nm, and then 3 reaction curves are drawn [19]. As a reference number, this article takes the A450nm value of the flat part of the maximum value on each curve. The data is written as [Ab]t. Three curves can be calculated to obtain three values. The values are [Aw]t, [Aw']t, and [Aw”]t, calculate Ka according to the following formula (Ka is the average value of K1, K2, and K3).

(8) $$\begin{array}{c} K_{a}=\frac{\left(n-1\right)}{2}\left(n\left[Aw^{\prime }\right]t-\left[Aw\right]t\right). \end{array}$$

In the formula, *n* = [Ag]t/[Ag′]t, [Ag]t, [Ag′]t represents the different concentrations of the original Pb2 + -ITCBE-BSA; [Aw]t, [Aw']t, [Aw”]t represents the mAb concentration corresponding to different concentrations of the original coating. Therefore, the calculation formula for the Ka value at the 3 coating concentrations corresponding to this experiment is

(9) $$\begin{array}{c} K_{1}=\frac{1}{2\left(2\left[Aw^{\prime }\right]t-\left[Aw\right]t\right)}, \end{array}$$

(10) $$\begin{array}{c} K_{2}=\frac{1}{2}\left(2\left[Aw^{\prime \prime }\right]t-\left[Aw^{\prime }\right]t\right), \end{array}$$

(11) $$\begin{array}{c} K_{3}=\frac{3}{2}\left(4\left[Aw^{\prime \prime }\right]t-\left[Aw\right]t\right). \end{array}$$

### 2.3. Gene Expression of Immune Infiltration

In this paper, the adjacency function is defined by weighting the similarity of gene expression profiles. This method only considers the association between two nodes in the network and cannot fully reflect the real situation inside the network [20]. Wrong adjacency relationships in the network will have a great impact on network topology inference. In order to reduce the influence of errors or sparse adjacency, it is more effective to use similarity measures based on interactive nodes or topological structures. In this paper, the genetic factors obtained by the topological overlap matrix in this study are genetic factors combined together in a comprehensive manner, which is biologically meaningful [21]. In an unauthorized network, the definition of topological overlap is

(12) $$\begin{array}{c} T_{qp}=\left\{\begin{array}{c} \frac{\sum_{u\neq p,q}a_{pu}a_{qu}+a_{pq}}{\min\left\{\sum_{u\neq p}a_{pu}-a_{pq},\sum_{u\neq q}a_{qu}-a_{pq}\right\}+1},\text{if }q\neq p\\ 1,\text{if }q=p \end{array}.\right. \end{array}$$

In a nonweighted network, ∑_u≠p,q_a_pu_a_qu_ represents the number of neighbor nodes connected to both node *p* and node *q*. ∑_u≠p,q_a_pu_a_qu_ represents the connectivity of node *p*. This formula can also be extended to weighted networks. Since 0≤≤1 in the weighted network, this paper can obtain

(13) $$\begin{array}{c} \underset{u\neq p,q}{\sum }a_{pu}a_{qu}\leq \underset{u\neq p}{\sum }a_{pu}-a_{pq}. \end{array}$$

And,

(14) $$\begin{array}{c} \underset{u\neq p,q}{\sum }a_{pu}a_{qu}\leq \underset{u\neq p}{\sum }a_{qu}-a_{pq}. \end{array}$$

Available at the same time,

(15) $$\begin{array}{c} \underset{u\neq p,q}{\sum }a_{pu}a_{qu}\leq \min\left\{\underset{u\neq p}{\sum }a_{pu}-a_{pq},\underset{u\neq q}{\sum }a_{qu}-a_{pq}\right\}. \end{array}$$

The numerator of the formula is ≤1, so the value in the weighted network is also in the interval [0,1]. The topological overlap matrix represents the similarity measure between nodes, and the degree of dissimilarity between nodes can be defined by

(16) $$\begin{array}{c} d_{pq}^{\omega }=1-T_{qp}. \end{array}$$

Using the index of dissimilarity between genes to cluster genes can obtain gene modules with higher specificity [22]. This paper conducts Venn analysis to narrow the scope of boot genes related to immune cells and stromal cells.

According to the topological overlapping structure of network nodes, this paper obtains the degree of dissimilarity between nodes and performs hierarchical clustering on this basis. For hierarchical clustering algorithms, the weighted average method is used to explain the relationship between variables, that is

(17) $$\begin{array}{c} d_{average}\left(clust.q1,clust.q2\right)=\frac{\sum_{p\in clust.q1}\sum_{p\in clust.q2}d_{p,\text{q}}}{\left|clust.q1\right|\left|clust.q2\right|}, \end{array}$$

where *d*_*p*,*q*_ represents the distance between classes *p* and *q*, and |clust.q1| and |clust.q2| represent the number of samples in classes *p* and *q*, respectively. This method makes full use of the information between variables and is one of the better methods in hierarchical clustering [23].

The single-sample gene enrichment analysis method enables the emergence of functionally relevant genomes based on gene discovery profile data analysis. According to the level of gene discovery, the algorithm first sorts all genetic factors to obtain the gene order [24]. After that, the concentration index of a certain gene is obtained by calculation.

(18) $$\begin{array}{c} ES\left(a,b\right)=\overset{n}{\underset{i=1}{\sum }}\left[P_{a}^{w}\left(a,b,i\right)-P_{nb}\left(a,b,i\right)\right],\text{where }P_{a}^{w}\left(a,b,i\right)=\underset{r\in a,j\leq i}{\sum }\frac{{\left|r_{j}\right|}^{\propto }}{\sum_{\text{r}\in a}{\left|r_{j}\right|}^{\propto }},\text{and }P_{nb}\left(a,b,i\right). \end{array}$$

()∑||/∑||∑(/())ES(*a*, *b*) is obtained by calculating the sum of the difference of the weighted empirical cumulative distribution function of all genes in genome *P*_*a*_^*w*^ and all remaining genes *P*_*nb*_. GSVA is a nonparametric unsupervised analysis method, mainly used to evaluate the gene set enrichment results of the chip nuclear transcriptome, so as to evaluate whether different pathways are enriched in different samples. In this study, the ssGSEA algorithm was used to obtain immune infiltration related data [25].

## 3. Experimental Results and Analysis

### 3.1. Functional Research of IGHG3

Malignant melanoma occurs on the skin and is one of the general malignant tumors of the skin. The incidence of this disease is lower than that of squamous cell carcinoma of the skin and basal cell carcinoma of the skin, but the degree of malignancy is significantly higher than the former two, and the incidence is gradually increasing, and there is a trend of younger development [26]. Malignant melanoma grows rapidly, has a high degree of invasion, and is prone to metastasis and recurrence.

This experiment first used four human melanoma cell lines, namely, A375, C918, MIC2C, and MIC2B cells, and cultured them with DMEM medium containing 10% fetal bovine serum and 100u/mL penicillin. All cell lines are kept in an incubator, and the culture environment is 5% CO2, 37°C.

Four types of human malignant melanoma cell lines were cultured in a 6-well plate. When the cell density was 80%, the four types of human malignant melanoma cells were collected. After waiting for the liquid in the culture solution to become transparent, add water to the tube before the dissolution is completed, and finally use the NanoDrop 2000c photometer to analyze and determine the concentration and quality of the liquid in the extraction culture solution.

The ΔCt of the 4 groups of melanoma cell lines in this experiment were A375 = 6.45, MUM − 2B = 8.51, MUM − 2C = 8.14, and C918 = 11.42. The PCR method is a DNA synthesis and amplification technology in vitro, which can quickly and specifically amplify any target DNA in vitro. It can be used for gene isolation and cloning, sequence analysis, gene expression regulation, gene polymorphism research, and many other aspects. It can be seen from the results of quantitative PCR that the four melanoma cells all express the IGHG3 gene in a high abundance, and the A375 cell line has the highest expression abundance, as shown in Figure 2. Therefore, this paper confirms that A375 cells are used for lentivirus infection.

This experiment is divided into an experimental group and a control group. The two groups follow the experimental procedures of cellular lentivirus infection [27]. 2*Δ*Ct reflects the relative expression level of IGHG3 gene in tumor cells of the control group and the experimental group. The 2*Δ*Ct of the two groups were experimental group =1.004 and control group =0.092. Quantitative PCR results showed that the expression of IGHG3 gene in A375 tumor cells in the control group was significantly inhibited at the mRNA level (*P* < 0.05), and the knockdown efficiency reached 85.6%. The details are shown in Figure 3.

The Celigo instrument was used to take pictures of tumor cells in the control group and the experimental group for 10 consecutive days, count the number of cells in the two groups, and draw a cell growth curve [28]. The results are recorded as Figure 4.

The number of tumor cells in the experimental group increased rapidly within 5 days, and the fluorescent cells covered the field of view on the 5th day. The number of fluorescent cells in the control group was significantly lower than that in the experimental group, and the number of fluorescent cells remained basically unchanged after 3 days.  Figure 5(a) shows the proliferation rate of tumor cells in the two groups, and Figure 5(b) shows the proliferation rate of tumor cells after excluding differences in plated cells. The conclusion is that the tumor cells of the experimental group are significantly lower than those of the control group, the cell proliferation of the experimental group is significantly inhibited, and the cell growth is slow after 3 days. Therefore, IGHG3 gene is involved in the regulation of A375 cell proliferation, and knocking out IGHG3 gene can inhibit melanoma cell proliferation [29].

It can be seen from Figure 5 that shRNA Ronchi virus will infect A375 cells after 5 days of culture. MTT is a yellow compound, a dye that accepts hydrogen ions, and can act on the respiratory chain in the mitochondria of living cells. Under the action of succinate dehydrogenase and cytochrome C, the tetrazolium ring splits to produce blue formazan crystals. The amount of formazan crystals produced is only proportional to the number of living cells. Then treated with MTT for 4 hours, it can be seen that the tumor cells of the experimental group and the control group proliferated in 1-4 days, but the proliferation rate of the experimental group was significantly lower than that of the control group, and the OD value of the experimental group was significantly lower than that of the control group. After 4 days, the OD value of the experimental group was smaller than that of the control group, and the proliferation of melanoma cells in the experimental group was significantly inhibited [30]. This is consistent with the results of Celigo cell count detection, indicating that knocking down IGHG3 has an inhibitory effect on cell proliferation. In this paper, the light absorption value of the blue-violet substance is detected by the instrument, and the number of living cells is positively correlated with the light absorption value. The detailed light absorption rate of the two groups is shown in Figure 6.

OD490 in the figure represents the number of viable cells.

### 3.2. Computational Mathematics Method to Detect the Influence of IGHG3 on A375

A375 positive cells were collected in the logarithmic proliferation phase, digested in routine, centrifuged, resuspended, and then counted to make the concentration of whole cells reach 0.75 × 10×/adjust to ml. A375 positive cells were seeded on 96-well plates, each well was 200 U1 or 1500 cells/well. Each cell group has 9 multibands, each cell is set with a zero adjustment hole (that is, only 20U1dmem complete medium is added), and 200ULBS is added to each well around the sampling hole. This plate method can also plant 296 plates.

Analyze the experimental data through SPSS statistical software, express the measured data as average ± standard deviation (x ± sd), and test the uniformity of dispersion. Through *t* test or *q* test, the methods are compared [31]. Check level *A* = 0.05. In *p* < 0.05, the difference is statistically significant: in *p* > 0.05, the difference is not statistically important. Comparing the in vitro invasion ability of the a375-negative cells of the control group and the blank control a375 cells, the difference between the two groups was not significant and statistically not significant (*p* = 0.174).

In order to test the effect of Highg3 on the discovery of A375 cells, A375 cells, A375 negative cells, and A375 positive cells were subjected to traditional centrifugation and washing [32]. In order to dissolve the cell lysate, extract the total protein of each cell, and detect the appearance of catechin protein in a375 cells, a375-negative cells, and a375-positive cells; western blot was used. In the blank control group, the proliferation activity of a375 cells was high, and the proliferation activity of A375-positive cells in the experimental group was significantly inhibited within 72 hours. The difference between the two groups is statistically significant. The detailed statistical results are shown in Table 1.

The results showed that the expression level of IGHG3 in A375-positive cells of the experimental group (0.44 ± 0.04) was significantly downregulated compared with the control group A375 cells (0.98 ± 0.09), down to 55.1%, and the difference was statistically significant. This shows that the lentiviral empty vector cannot significantly affect the expression and output of *β*-catenin protein in A375 cells. The results are shown in Figure 7(a). The colonies formed by A375 cell clones in the blank control group were larger, and the colonies formed by cells in the A375-positive group were smaller, and the number of colonies formed was less (55.00 ± 15.34). The clone completion rate was 27.50% ± 7.67%. Compared with the A375-feminine group, *P* < 0.05; compared with the A375 group, *P* < 0.05. The result is shown in Figure 7(b).

It can be seen from Figure 7 that in the blank control group, the in vitro invasion ability of A375 cells is strong, and the in vitro invasion ability of A375 positive cells in the experimental group is inhibited. The difference between the two groups is statistically significant. The in vitro invasion ability of A375 negative cells in the negative control group is also very high [33]. Compared with the in vitro invasion ability of A375-positive cells in the experimental group, the cell invasion ability is significantly different, which is statistically important.

In this experiment, this article uses a floating control sub-G1 peak method for detecting intracellular death. The basic principle is that in apoptosis cells, the nucleotides at the end of the cell are activated to initiate programmed suicide cells. Since the DNA chain is cut between the nucleotides, the DNA as a unit is broken down into fragments by the nucleotides. These small DNA fragments are released from the nucleus, and the DNA content in the cells is lower than that of normal cells. Use floating cells to analyze the DNA content of the cells. If the amount of DNA in the g1 nucleus is less than that of the cells, other cells will form before the gl peak. One peak (sub-G1 peak or SUBG1 peak) is considered to be a dead cell. The death rate of A375 cells in the blank control group was 3.14 ± 0.41%, and the death rate of A375-positive cells in the experimental group was significantly increased (18.51 ± 2.15%). There is a clear gap between the two. In the negative control group, the death rate of A375 negative cells was 4.02 ± 0.36%, which was not significantly different from the death rate of A375 cells in the blank control group. In the negative control group, the Apollo rate of A375-negative cells was significantly different from the A375-positive cells of the experimental group [34]. The details are recorded in Table 2.

The lentiviral vector used in this experiment carries a small RNA with interfering fragments and infects human malignant melanoma A375 cells. The Ronchi virus carries the genetic factor of the green fluorescent protein, and after successful infection, it will show green fluorescence to the host cell. At the same time, after the wrench virus infects the host cell, the target gene fragment is fused with the host gene and then transmitted to the descendant cells together with the cell replication to form a stable infected cell strand. By observing the ratio of green fluorescent cells and analyzing the transmission efficiency of the western barrier, it was verified whether the interference of high g3 expression was successful. Excessive cell proliferation is one of the reasons for the malignant increase of malignant melanoma. Experimental results show that the transmission rate of A375 cells is greater than 70% under an inverted fluorescence microscope. Western blot results showed that the expression of IGHG3 in A375-positive cells was significantly downregulated compared to A375 cells in the blank control group, reaching 55.1%; the expression of IGHG3 in A375-feminine cells infected with empty lentivirus was not significantly different from that in A375 cells. It can be considered that the use of IGHG3 in this experiment successfully interfered with the reproduction of melanoma cells.

### 3.3. Infiltrating Immune Cells of Melanoma

Based on the above research situation, this study used tumor cells to express immune cells infiltrating the melanoma microenvironment at the tissue level, such as regulatory T lymphocytes and various parts of melanoma, in order to explore the characteristics of related cytokines. This article will jointly evaluate the relationship between these two cytokines and regulatory T lymphocyte infiltration, analyze their differences in different molecular types of invasive melanoma, and explore the prognostic significance of the two cytokines in patients with melanoma in advance. In the tumor microenvironment, the proportion of immune cells (such as B cells and T cells) derived from the bone marrow depends on the type of tumor. As shown in Figure 8, different immune cells have different immune responses to tumors.

Among them, T-helper-1 cells, natural killer cells, M1 phenotype maclovac and DC1 phenotype dendritic cells hinder tumor formation and development. On the other hand, T-helper 2 cells, M2 maclovac, and DC2 dendritic cells and regulatory T cells (Treg) suppress the immune response and promote the generation and development of tumors. Factors secreted by different immune cells, such as tumor growth factor, vascular growth factor (VEGF), angioside, FGF2, silicone, IL-6, and IL-10, break down the matrix that inhibits receptors and promotes the appearance of immune cells. In ovarian cancer and colorectal cancer, the high incidence of proangiogenic factors reduces the infiltration of th1/cd8+ T cells. The high detection of TGF*β* weakened the activation, maturation, and differentiation of cd4 + t cells, cd8 + t cells, natural killer cells, dendritic cells, neutrophils, and maclovac. Among them, CD8 T cells can recognize and kill the immune cells of melanoma cells, which are considered to have the potential to eradicate tumors.

In short, the immune system has immunoediting effects on tumor cells at different stages of tumor formation and development. Different immune cells and growth factors in the tumor microenvironment can inhibit or promote the growth and development of tumors, forming a complex immune response. The cell's TGF*β* factor becomes an abnormal functional state and gradually loses the ability to recognize and attack tumor cells. A detailed understanding of the unique properties of different immune cells can open up new treatment methods for cancer immunotherapy. In this paper, the 9 immune cell data from ENCODE are used to construct the gene regulation network of each cell. This article compares and analyzes 9 immune cell genes of normal people.  Table 3 shows the specific genes of each cell among the genetic factors shared by different cell types and different cells.

Through comparative analysis and the establishment of a transfer factor regulation network with 9 immune cells, it is found that there are 32 common transfer factors, and each cell has a specific transfer factor. B cells have 168 transfer factors and 14 specific transfer factors. CD4+ T cells have two specific transfer factors ASCL2, Borcs8-MEF2b's 164 transfer factor, CD8+ T cells have 161 transfer factors, and an uneven transfer factor MEIS1-AS3, of which dc cells have 254 transfer factors and 31 specific transfer factors. NK cells have 129 transcription factors, and one specific transcription factor is TBX3. There are 143 transcription factors in regulatory T cells and one specific transcription factor ESX1. T-helper-17 has 217 transcription factors and 84 specific transcription factors. T-helper-1 has 119 transcription factors, and one specific transcription factor is NR2C2. T-helper-2 has 160 transcription factors and 1 specific transcription factor OTX1.

The experiment initially found that the characteristics of lncRNA CYTOR were significantly different in black tumor samples. In addition, the analysis of the survival curve in Figure 9 shows that its high performance is significantly associated with poor prognosis.

Computational mathematics is a general algorithm for studying immune infiltration. The gene expression results obtained by RNA-Seq or gene chip can evaluate the results of tumor interstitial cell and immune cell infiltration, which can be used to study the immune infiltration between different samples. The results are shown in Table 4.

Next, using stromal score and immune cell data, the box plot shown in Figure 10 was created, and it was found that the expression level of CYTOR was significantly correlated with the immune fusion score.

IGHG3 is significantly reduced in human and mouse CD8+ T cells with abnormal function, while the abnormal function marker genes Pdcd1 and Ctla4 are significantly increased. Increasing IGHG3 can significantly reduce the expression of Pdcd1, Ctla4, and Zfx genes, restore the function of abnormal CD8+ T cells, and extend the survival period of patients with melanoma models, which may become a potential treatment.

The results showed that in the tumor microenvironment, the expression of CD7 and P4HB surface receptors on tumor-invasive dysfunctional CD8+ T cells (PD1) was shut down, while the expression of GMEB2 transcription factor shut down by dysfunctional CD8+ T cells and the two cell surface receptors were shut down. There is no direct regulatory relationship in the body, and there may be other modes of action such as miRNA that cause the expression of these two cell surface receptors to be closed. As long as the treatment is timely and appropriate treatment is used, the survival rate of melanoma patients over five years can reach more than 90%.

In summary, as a tumor suppressor gene, IGHG3 can reduce the expression of CD8+ T cells and melanoma cells with melanin-infiltrating dysfunction in humans and mice. DIG3 can act on insufficient CD8+ T cells and melanoma cells.

## 4. Conclusion

The immune microenvironment of tumors is very complex and may be related to different types of cells. This relationship changes at all stages of tumor development. The results of this analysis show that the strongest positive correlation between melanoma is the good mid-ball and activated obese cells, and the strongest negative correlation is between cd8 + t cells and m0 cells. The relationship between immune cells is not yet clear. In future research, the relationship needs to be further studied. Predicting these potential correlations can be used to fight infection and cancer.

The composition of infiltrating immune cells in melanoma is different, and different infiltration characteristics may affect the prognosis of patients, which helps people to develop more effective treatments. The experimental results showed that after shRNA lentivirus infection, the detection of IGHG3 gene expression through computational mathematical methods had a significant inhibitory effect on A375 cells in the experimental group, and the knockdown efficiency reached 85.6%.

## Figures and Tables

**Figure 1:** Material exchange relationship between cells in IGHG3 treatment.

**Figure 2:** Expression abundance of IGHG3 gene in 4 melanoma cell lines.

**Figure 3:** IGHG3 gene reduction in A375 tumor cells after lentivirus infection.

**Figure 4:** Results of tumor cell changes in the two groups.

**Figure 5:** The curve of the number of cells infected by the virus over time in the two groups.

**Figure 6:** Comparison of the light absorption rate of the two groups over time.

**Figure 7:** The effect of IGHG3 on the expression of *β*-catenin protein and the ability of clone formation in A375 cells.

**Figure 8:** Immune cells in the microenvironment play a role in hindering or promoting the production of tumor cells.

**Figure 9:** Survival curves of melanoma in two cases.

**Figure 10:** Box plot of stromal score and immune score.

**Table 1:** Computational mathematics detection of the effect of IGHG3 on the proliferation activity of A375 cells.

Time	A375	A375-feminine	A375-positive
12 h	0.1667 ± 0.0417	0.2379 ± 0.0788 △	0.2084 ± 0.0703 ∗
24 h	0.2368 ± 0.0369	0.3722 ± 0.0653 △	0.2787 ± 0.0603 ∗
36 h	0.3591 ± 0.0542	0.4875 ± 0.0377 △	0.4137 ± 0.0847 ∗
48 h	0.4711 ± 0.0574	0.5826 ± 0.09 △	0.4974 ± 0.0201 ∗
60 h	0.5745 ± 0.0389	0.722 ± 0.0643 △	0.6157 ± 0.0556 ∗
72 h	0.6609 ± 0.0427	0.831 ± 0.0728 △	0.6907 ± 0.0245 ∗

△: Compared with the blank control group, *P* > 0.05.

∗: Compared with the negative control group, *P* < 0.05.

**Table 2:** Flow cytometry to detect the effect of IGHG3 on A375 cell apoptosis.

Group	Sub G1 period (%)	*P*
A375	3.14 ± 0.41	<0.05
A375-feminine	4.02 ± 0.36△	>0.05
A375-positive	18.51 ± 2.15∗	<0.05

**Table 3:** Comparative analysis of various immune cell gene regulatory networks.

Cell type	Annotated gene	Specific gene
NK	11130	1155
B	7476	903
CD4+	7005	310
CD8+	12310	96
DC	7483	308
T-HELPER-1	11372	697
T-HELPER-2	7853	355
T-HELPER-17	8480	505
REGULATORY	7927	486

**Table 4:** Each score of the sample.

	Stromal score	Immune score	ESTIMAT score	Tumor purity
1	-1559.1	-665.9	890.5	0.78
2	-1261.7	-524	-2306	0.9
3	-1167.2	-145.8	633	0.81
4	-170.8	813.1	-844.6	0.8
5	-1050.6	178.6	1554.4	0.89
6	-1230	-36.8	1546.4	0.89
7	-112.4	-660.2	513.4	0.78
8	-1553.4	-236.9	-153.8	0.78
9	150	-145.3	-597.8	0.81
10	213.8	259.1	-1774.5	0.83
11	-1120.6	-116.6	-1276.3	0.77
12	-728.5	-655.6	-2440.8	0.78
13	-336.7	-762.9	-1684.6	0.81
14	-1388.1	-714.3	818.3	0.77
15	-943.6	87	648	0.78

## Data Availability

The data used to support the findings of this study are available from the corresponding author upon request.
